# Selective Molecular Alterations in the Autophagy Pathway in Patients with Lewy Body Disease and in Models of α-Synucleinopathy

**DOI:** 10.1371/journal.pone.0009313

**Published:** 2010-02-19

**Authors:** Leslie Crews, Brian Spencer, Paula Desplats, Christina Patrick, Amy Paulino, Edward Rockenstein, Lawrence Hansen, Anthony Adame, Douglas Galasko, Eliezer Masliah

**Affiliations:** 1 Department of Pathology, University of California San Diego, La Jolla, California, United States of America; 2 Department of Neurosciences, University of California San Diego, La Jolla, California, United States of America; University of Nebraska Medical Center, United States of America

## Abstract

**Background:**

Lewy body disease is a heterogeneous group of neurodegenerative disorders characterized by α-synuclein accumulation that includes dementia with Lewy bodies (DLB) and Parkinson's Disease (PD). Recent evidence suggests that impairment of lysosomal pathways (i.e. autophagy) involved in α-synuclein clearance might play an important role. For this reason, we sought to examine the expression levels of members of the autophagy pathway in brains of patients with DLB and Alzheimer's Disease (AD) and in α-synuclein transgenic mice.

**Methodology/Principal Findings:**

By immunoblot analysis, compared to controls and AD, in DLB cases levels of mTor were elevated and Atg7 were reduced. Levels of other components of the autophagy pathway such as Atg5, Atg10, Atg12 and Beclin-1 were not different in DLB compared to controls. In DLB brains, mTor was more abundant in neurons displaying α-synuclein accumulation. These neurons also showed abnormal expression of lysosomal markers such as LC3, and ultrastructural analysis revealed the presence of abundant and abnormal autophagosomes. Similar alterations were observed in the brains of α-synuclein transgenic mice. Intra-cerebral infusion of rapamycin, an inhibitor of mTor, or injection of a lentiviral vector expressing Atg7 resulted in reduced accumulation of α-synuclein in transgenic mice and amelioration of associated neurodegenerative alterations.

**Conclusions/Significance:**

This study supports the notion that defects in the autophagy pathway and more specifically in mTor and Atg7 are associated with neurodegeneration in DLB cases and α-synuclein transgenic models and supports the possibility that modulators of the autophagy pathway might have potential therapeutic effects.

## Introduction

Alzheimer's disease (AD) and Parkinson's disease (PD) are the most common causes of dementia and movement disorders in the elderly [1], [2]. While progressive accumulation of Aβ dimers and oligomers has been identified as one of the central toxic events in AD leading to synaptic dysfunction [3], [4], accumulation of α-synuclein (α-syn) resulting in the formation of oligomers has been linked to the pathogenesis of PD [5], [6], [7], [8], [9].

The pathology of AD and PD overlap in a heterogeneous group of conditions denominated jointly Lewy body disease (LBD) [10], [11], [12], [13], [14]. While in patients with dementia with Lewy bodies (DLB) the clinical presentation is of dementia followed by parkinsonism, in patients with PD dementia (PDD) the initial signs are of parkinsonism followed by dementia [15], [16], [17], [18]. In DLB, Aβ promotes α-syn aggregation and toxicity *in vivo* [19], and Aβ and α-syn might directly interact [20] to form hybrid channel like structures [21].

Alterations in the rate of synthesis, aggregation and clearance of these proteins might be responsible for the formation of toxic Aβ and α-syn oligomers in DLB [22]. Impaired clearance of the α-syn aggregates might play an important role in the pathogenesis of PD and DLB [23], [24]. Among the lysosomal pathways involved, the autophagy signaling cascade has emerged as a key mechanism for the removal of α-syn aggregates. Autophagy is the major pathway involved in the degradation of long-lived proteins and organelles, cellular remodeling, and survival during nutrient starvation [25], [26]. There are three distinct autophagic pathways [27], [28]: i) macroautophagy, ii) microautophagy and iii) chaperone-mediated autophagy (CMA). Autophagy has been linked to neuronal cell death [29], [30] and is abnormally activated in mouse models of neurodegeneration and in neurodegenerative disorders such as AD, PD and Huntington's disease (HD) [31], [32]. Macroautophagy is constitutively active and highly efficient in healthy neurons and recent studies indicate that the autophagic pathology observed in AD most likely arises from impaired clearance of autophagic vacuoles (AVs) rather than strong autophagy induction alone [33] suggesting selective alterations in molecular components of the autophagy pathway. For example, in the brains of patients with AD, levels of the AV protein Beclin-1 are severely down modulated [34].

In PD recent studies have suggested that α-syn aggregates might interfere with the autophagy mechanisms and lead to neurodegeneration [23], [35], [36], [37], [38], [39]. Mutant forms of α-syn found in familial PD patients [23] as well as oxidized forms of α-syn [40] found in sporadic PD and DLB have been shown to block autophagy, and a-syn contains a consensus sequence for CMA targeting. In neuronal cell cultures [41] and in transgenic (tg) mice, α-syn overexpression is associated with impaired autophagy and neurodegeneration that is reversed by Beclin-1 [42]. Further supporting a role for lysosomal dysfunction in LBD, previous studies have shown that in lysosomal storage disorders such as Gaucher disease [43], [44] and Niemann-Pick disease [45], there is increased susceptibility to develop parkinsonism and α-syn accumulation.

Taken together, these lines of evidence suggest that in DLB and PD, specific molecular defects in the autophagy pathway might play a role in the pathogenesis of these disorders. In this context, the main objective of the present study was to investigate alterations in components of the autophagy pathway in DLB and in a-syn tg models. We found that levels of mTor were increased and Atg7 levels were reduced in the brains of patients with DLB and a-syn tg mice. Moreover, activating autophagy by rapamycin treatment or viral-mediated delivery of Atg7 ameliorated a-syn accumulation and the related neuropathology. This supports the notion that alterations in the autophagy pathway play a role in DLB/PD and supports the possibility that modulators of the autophagy pathway might have potential therapeutic effects.

## Materials and Methods

### Ethics Statement

This study was conducted according to the principles expressed in the Declaration of Helsinki. For studies utilizing human tissues, all tissues were obtained from the University of California, San Diego Alzheimer's Disease Research Center (ADRC). Written informed consent for neurobehavioral evaluation, autopsy, and for the collection of samples and subsequent analysis was obtained from the patient and caregiver (usually the next of kin) before neuropsychological testing and after the procedures of the study had been fully explained. The study procedures conformed to Federal guidelines for the protection of human subjects and were reviewed and approved by the UCSD Institutional Review Board. For animal studies, all animals were handled in strict accordance with good animal practice and all procedures were completed under the specifications set forth by the UCSD Institutional Animal Care and Use Committee.

### Cases and Neuropathological Evaluation

The study included a total of 24 cases (Table 1); of them, 6 were non-demented controls, 12 were DLB cases and the other 6 were AD cases. For the present study we chose to focus on DLB because of its frequency and widespread accumulation of a-syn in neocortical and limbic structures [46], [47], [48]. Autopsy material was obtained from patients studied neurologically and psychometrically at the UCSD ADRC. At autopsy, brains were divided sagittally, and samples from the left mid temporal cortex were fixed in 4% paraformaldehyde (PFA) and sectioned at 40 µm for immunocytochemical analysis. Frozen samples from the right were used for immunoblot analysis. The temporal cortex was selected because previous studies have shown considerable pathology and accumulation of α-syn in this region in patients with DLB [47], [48], [49].

**Table 1:** Summary of clinico-pathological characteristics.

Diagnosis	N =	Mean Age (yrs)	Mean brain weight	Gender M/F	Mean PMT (hrs)	Mean Duration (yrs)	Blessed score	Frontal cortex Amyloid Plaques (0.1sq mm)	Temporal cortex Lewy bodies (0.1sq mm)
Control	6	79.8±2	1150±115	4/2	6.5±2	NA	0–1	0	0
AD	6	81±1	1058±97	3/3	8±1	12.8±1	19–33	50	0
DLB	12	82.7±2	1074±119	4/8	7.2±1.5	9.8±	5–32	33	12±2

For routine neuropathological diagnosis, paraffin sections from neocortical, limbic and subcortical regions were stained with haematoxylin and eosin (H&E) or thioflavine-S [50], [51], and Braak stage was assessed [52]. Based on previously published clinical and pathological findings [53], cases were subdivided into: 1) non-demented age-matched controls, 2) AD cases, and 3) DLB cases. All cases met the Consortium to Establish a Registry for AD (CERAD) and National Institute of Aging (NIA) criteria for diagnosis and displayed neuritic plaques and tangle formation in the neocortex and limbic system [12], [54]. The diagnosis of DLB was based on the clinical presentation of dementia and the pathological findings of LBs in the locus coeruleus, substantia nigra (SN), or nucleus basalis of Meynert, as well as in cortical regions. LBs were detected using H&E stain or anti-ubiquitin and anti-α-syn antibodies as recommended by the Consortium on DLB criteria for a pathologic diagnosis of DLB [12]. In addition to the presence of LBs, the great majority of these cases displayed sufficient plaques and tangles to be classified as Braak stages III–IV. Specifically, DLB cases had abundant plaques in the neocortex and limbic system but fewer tangles compared to AD cases.

### a-Synuclein Transgenic Mice and Treatments

For this study, heterozygous tg mice (Line D) expressing human wildtype α-syn under the regulatory control of the PDGFβ promoter [55] were used. These animals were selected because they display abnormal accumulation of detergent-insoluble α-syn in the neocortex and limbic system and develop α-syn-immunoreactive inclusion-like structures in the brain [56]. Although some nuclear staining has been observed in this model, distinct cytoplasmic inclusion-like structures have been consistently identified by confocal and electron microscopy [19], [55], [56], [57]. Furthermore, these animals also display neurodegenerative and behavioral deficits that mimic certain aspects of DLB. For western blot and immunocytochemical studies levels of components of the autophagy pathway were compared to littermate non tg controls and to an APP tg model (line J9M) of AD-like pathology. These mice express human APP 770/751 and 695 under the PDGFβ promoter [58].

Additional experiments with the α-syn tg mice included treatments with the autophagy activator rapamycin (Sigma-Aldrich, St. Louis, MO). Because rapamycin poorly crosses into the CNS, it was infused intra-cerebrally into the lateral ventricle of 9-month old mice at a concentration of 20mg/kg. Briefly as previously described [59], mice were anesthetized and under sterile conditions a 26 gauge stainless steel cannula was implanted stereotaxically into the lateral ventricle using the bregma as a reference (Franklin and Paxinos, bregma 0.5mm; 1.1mm lateral; depth 3mm) and secured to the cranium using superglue. The cannula was connected via a 5 mm coil of V3 Biolab vinyl to a model 1007D osmotic minipump (Alzet, Cupertino, CA) surgically placed subcutaneously beneath the shoulder. The solutions were delivered at a flow rate of 0.5ul per hour for 2 weeks. The pump was left for an additional 2 weeks and mice were euthanized one month after the initiation of the infusions. Brains were removed and divided sagittally. One hemibrain was postfixed in phosphate-buffered 4% PFA, pH 7.4, at 4°C for 48 h and sectioned at 40 µm with a Vibratome 2000 (Leica, Nussloch, Germany) and placed in cryosolution, while the other hemibrain was snap frozen and stored at −70°C for RNA and protein analysis.

### Construction of Lentiviral Vectors and Injection of LV-Atg7 into α-Synuclein Transgenic Mice

The mouse Atg7 cDNA (Open Biosystems, Huntsville, AL) was PCR amplified and cloned into the third generation self-inactivating lentivirus vector (LV) [60] with the CMV promoter driving expression. Lentiviruses expressing α-syn, Atg7, luciferase, shAtg7, GFP, shLuciferase, or empty vector (as controls) were prepared by transient transfection in 293T cells [60], [61]. The empty LV contained the viral genome with the CMV promoter, with no gene inserted downstream of the promoter.

A total of 12 α-syn tg mice from line D (9 months old) were injected with 3 µl of the LV preparations (2.5×10^7^ TU) into the temporal cortex and hippocampus (using a 5 µl Hamilton syringe). Briefly, as previously described [62], mice were placed under anesthesia on a Koft stereotaxic apparatus and coordinates (hippocampus: AP −2.0 mm, lateral 1.5 mm, depth 1.3 mm and cortex: AP −.5 mm, lateral 1.5 mm, depth 1.0 mm) were determined as per the Franklin and Paxinos Atlas. The LVs were delivered using a Hamilton syringe connected to a hydraulic system to inject the solution at a rate of 1 µl every 2 min. To allow diffusion of the solution into the brain tissue, the needle was left for an additional 5 min after the completion of the injection. Mice received unilateral injections (right side) to allow comparisons against the contralateral side, with either LV-Atg7 (n = 6), or LV-control (n = 6). Additional controls were performed by injecting non tg littermates with either LV-Atg7 (n = 6), or LV-control (n = 6). Mice survived for 1 month after the lentiviral injection. As an additional control for LV injection, age matched littermates were injected with LV-luciferase. Since no differences were observed between the LV-control and the LV-luciferase, all data presented here are shown with the LV-control vector.

Following NIH guidelines for the humane treatment of animals, mice were anesthetized with chloral hydrate and flush-perfused transcardially with 0.9% saline. Brains and peripheral tissues were removed and divided sagittally. The right hemibrain was post-fixed in phosphate-buffered 4% PFA (pH 7.4) at 4°C for 48 hours for neuropathological analysis, while the left hemibrain was snap-frozen and stored at −70°C for subsequent RNA and protein analysis.

### Cell Culture and Treatments

For *in vitro* experiments we used the previously described rat neuroblastoma cell line B103 [63]. This model was selected because overexpression of α-syn in these cells interferes with neuronal plasticity (reduced neurite outgrowth and adhesion) but does not result in overt cell death [63], [64]. This model mimics the early pathogenic process of PD where cell death is preceded by reduced neurite outgrowth and synaptic alterations. For all experiments, cells were plated in complete media (DMEM [Invitrogen, Carlsbad, CA] supplemented with 10% FBS (Irvine Scientific, Santa Ana, CA) and infected with LVs expressing α-syn, Atg7, shAtg7, or controls at a multiplicity of infection (MOI) of 40. After infection, cells were incubated for 48 hr in a humidified 5% CO_2_ atmosphere at 37°C. All experiments were conducted in triplicate to ensure reproducibility.

To investigate whether LC3 levels are modulated by α-syn or Atg7 over-expression or knockdown, LC3 levels were analyzed in coverslips with LC3-GFP. B103 cells were grown as described above and were then plated onto poly L-lysine coated glass coverslips at a density of 5×10^4^ cells. Five hours after plating, cells were infected with the LV-αsyn and/or LV-Atg7 or LV-shAtg7 (or controls) and incubated for 48 hours. All coverslips were also co-infected with an LV expressing LC3-GFP at an MOI of 40. Cultures were then washed 2× with serum-free DMEM and then fed either complete media or serum-free media for 12 hours before fixation with 4% PFA. Briefly as previously described [34], coverslips were treated with Prolong Gold antifading reagent with DAPI (Invitrogen) and imaged with the LSCM to determine the number of GFP-positive granular structures consistent with autophagolysosomes using semiautomatic image analysis system and the ImageQuant software. For each condition an average of 50 cells were analyzed.

### Antibodies

For western blot and immunohistochemical analysis of the autophagy pathway, polyclonal antibodies against mTor (1∶1000, Sigma); phosphorylated-mTor (p-mTor, 1∶1000, Cell Signaling Technology, Beverly, MA); Atg5 (1∶1000, Abcam, Cambridge, MA); Atg6 or Beclin-1 (1∶1000, Novus Biologicals, Littleton, CO); Atg7 (1∶500, Abcam); Atg8 or LC3 (1∶1000, Abcam); Atg10 (1∶500, Abcam); Atg12 (1∶1000, Abcam); Cathepsin D (1∶500, Calbiochem, San Diego, CA). Detection of α-syn was performed with a rabbit polyclonal (1∶500, Millipore, Temecula, CA) and a mouse monoclonal antibody (1∶500, clone syn211, Sigma).

### Immunohistochemistry, Image Analysis and Laser Scanning Confocal Microscopy

Briefly, as previously described [65], free-floating 40 µm thick vibratome sections were washed with Tris buffered saline (TBS, pH 7.4), pre-treated in 3% H_2_O_2_, and blocked with 10% serum (Vector Laboratories, Burlingame, CA), 3% bovine serum albumin (Sigma), and 0.2% gelatin in TBS-Tween (TBS-T). For human brains, sections from the temporal cortex were used; for the mice sagittal sections from the complete brain were studied. Sections were incubated at 4°C overnight with the primary antibodies. Sections were then incubated in secondary antibody (1∶75, Vector), followed by Avidin D-horseradish peroxidase (HRP, ABC Elite, Vector) and reacted with diaminobenzidine (DAB, 0.2 mg/ml) in 50 mM Tris (pH 7.4) with 0.001% H_2_O_2_. Control experiments consisted of incubation with pre-immune rabbit serum. To investigate the effects of postmortem delay and fixation on the levels of mTor immunoreactivity, preliminary studies were performed in a subset of cases (n = 5) with postmortem delay ranging from 4–48 h.

Immunostained sections were imaged with a digital Olympus microscope and assessment of levels of mTor, Atg7, LC3 and Cathepsin D immunoreactivity was performed utilizing the Image-Pro Plus program (Media Cybernetics, Silver Spring, MD). For each case a total of three sections (10 images per section) were analyzed in order to estimate the average number of immunolabeled cells per unit area (mm^2^) and the average intensity of the immunostaining (corrected optical density).

Double-immunocytochemical analyses was performed utilizing the Tyramide Signal Amplification™-Direct (Red) system (NEN Life Sciences, Boston, MA). Specificity of this system was tested by deleting each primary antibody. For this purpose, sections were double-labeled with the monoclonal antibodies against α-syn (1∶20,000, Cell Signaling) detected with Tyramide Red, and either mTor, Cathepsin D or LC3 detected with fluorescein isothiocyanate (FITC)-conjugated secondary antibodies (1∶75, Vector).

All sections were processed simultaneously under the same conditions and experiments were performed twice for reproducibility. Sections were imaged with a Zeiss 63X (N.A. 1.4) objective on an Axiovert 35 microscope (Zeiss, Germany) with an attached MRC1024 laser scanning confocal microscope (LSCM) system (BioRad, Hercules, CA).

### Analysis of Neurodegeneration

To evaluate the integrity of the dendritic system, blind-coded 40µm-thick vibratome sections from mouse brains fixed in 4% PFA were immunolabeled with the mouse monoclonal antibody against microtubule associated protein 2 (MAP2) (dendritic marker, 1∶40, Millipore), as previously described [66]. After an overnight incubation with the primary antibody, sections were incubated with FITC-conjugated horse anti-mouse IgG secondary antibody (1∶75, Vector), transferred to SuperFrost slides (Fisher Scientific, Tustin, CA) and mounted under glass coverslips with anti-fading media (Vector). All sections were processed under the same standardized conditions. The immunolabeled blind-coded sections were imaged with the LSCM (MRC1024, Bio-Rad) and analyzed with the Image 1.43 program (NIH), as previously described [66], [67].

### Western Blot Analysis

Immunoblot analysis was performed as previously described [68]. Briefly, brain homogenates (temporal cortex for human tissues and cortex for mice) or cultured cells were solubilized in lysis buffer (1% Triton X-100, 10% glycerol, 50 mM HEPES, pH 7.4, 140 mM NaCl, 1mM EDTA, 1mM Na_3_VO_4_, 20 mM β-glycerophosphate, and proteinase inhibitor cocktails). Brain homogenates were separated into cytosolic and membrane fractions by centrifugation at 100,000×g for 1 hr at 4C. Isolation of lysosomal fractions from brain tissue was performed by differential centrifugation in a sucrose-based buffer essentially as previously described [69]. Briefly, tissues were minced with a razor blade and homogenized in ice-cold 50 mM Tris/HCl buffer, pH = 7.4, containing 0.25 M sucrose, 10 mM EDTA, 3 mM MgCl_2_, with protease and phosphatase inhibitor cocktails (Calbiochem) added fresh (sucrose/Tris buffer). After filtration through a mesh to remove cell debris and capsular fragments, the homogenate was centrifuged at 1000 g for 5 min to obtain the nuclear fraction (pellet 1, P1). The supernatant was centrifuged again at 10,000 g for 10 min to collect the mitochondrial fraction (pellet 2, P2). The resulting supernatant was centrifuged at 20,000 g for 10 min to obtain the lysosomal fraction (pellet 3, P3). Finally, the supernatant remaining after the removal of the lysosomal fraction was centrifuged at 180,000 g for 30 min to separate the microsomal fraction (pellet 4, P4) from the cytosol/extracellular fluid fraction (supernatant 4, S4). Pellets were gently resuspended in 0.25 mL sucrose/Tris buffer, and all fractions were stored at −80°C until further processing.

For western blot analysis, 20 µg of each fraction was resolved by SDS-PAGE on 4–12% Bis-Tris gels (Invitrogen) and electroblotted onto Immobilon membranes (Millipore). The membranes were blocked with phosphate-buffered saline (PBS) with 0.2% Tween-20 (PBST) containing 3% skim milk or bovine serum albumin (BSA), followed by incubation with primary antibodies in PBST containing 5% BSA. After washing with PBS, the membranes were incubated with rabbit anti-mouse secondary antibodies (1∶5000, American Qualex, San Clemente, CA) and visualized with enhanced chemiluminescence (ECL, PerkinElmer, Wellesley, MA) and analyzed with the VersaDoc gel imaging system (BioRad).

### Electron Microscopy

Briefly, as previously described [42], vibratome sections from control, DLB brains and α-syn tg mice were post-fixed in 1% glutaraldehyde, then treated with osmium tetraoxide and embedded in epon araldite. Once the resin hardened, blocks were sectioned with an ultramicrotome (Leica). Grids were analyzed with a Zeiss OM 10 electron microscope as previously described [70]. Micrographs from pyramidal neurons in the temporal cortex were randomly acquired from 3 grids, and electron micrographs were acquired at a magnification of 25,000 each.

### Statistical Analysis

All experiments were conducted in triplicate on blind-coded samples. After the results were obtained, the code was broken and data were analyzed with the StatView program (SAS Institute, Inc., NC). Comparison among groups of expression levels of components of the autophagy pathway were performed by one-way ANOVA with post-hoc Dunnett's or Tukey-Kramer. All results are expressed as mean ± SEM.

## Results

### Alterations in the Levels of mTor and Atg7 Are Associated with Lysosomal Alterations the Brains of DLB Patients

Recent evidence suggests that impaired functioning of the lysosomal pathways (eg: autophagy) involved in α-syn clearance might play a role in the pathogenesis of DLB [23], [24]. For this reason, expression levels of members of the autophagy pathway were analyzed in the temporal cortex of control, AD and DLB patients. By immunoblot analysis, mTor was identified as a triplet band at an estimated molecular weight of 280–290 kDa that was more abundant in the membrane than in the cytosolic fraction (Figure 1A, B). Compared to non-demented controls and AD cases, levels of mTor and phosphorylated-mTor (p-mTor) were elevated in the brains of DLB cases (Figure 1A, C). In both the membrane and cytosolic fractions Atg7 was identified as a doublet at an estimated molecular weight of 78 kDa (Figure 1A, B). In DLB cases, levels of Atg7 were moderately reduced compared to controls and AD cases (Figure 1A, D). No differences were observed between controls and AD cases (Figure 1A, D). Other components of the autophagy pathway such as Atg5 (32 kDa) and Atg12 (20kDa) were identified as single bands that were more abundant in the membrane than in the cytosolic fractions (Figure 1A, B). No differences were detected among the 3 groups in the levels of these Atg proteins (Figure 1A, D). Beclin-1 was detected as a single band at 50 kDa that was more abundant in the membrane than the cytosolic fraction (Figure 1A, B). Consistent with previous studies [34], levels of Beclin-1 in the membrane fractions were reduced in the AD cases compared to non-demented controls and DLB, however no differences in Beclin-1 levels were detected between non-demented controls and DLB cases (Figure 1A, C).

**Figure 1:** Immunoblot analysis of the autophagy pathway in the brains of AD and DLB patients. Brain homogenates from the temporal cortex of non-demented controls, AD, and DLB patients were separated into membrane and cytosolic fractions, and 20 µg of each sample was subjected to gel electrophoresis. Immunoblots were probed with antibodies against mTor, phosphorylated (p) mTor, Beclin-1, Atg5, Atg7, Atg12 and Actin. (A) Representative immunoblots of membrane fractions. (B) Representative immunoblots of cytosolic fractions. (C) Semi-quantitative analysis of levels of mTor, p-mTor, and Beclin-1 in membrane fractions from the brains of control, AD and DLB patients. Levels of mTor were significantly increased in DLB patients. (D) Semi-quantitative analysis of levels of Atg5, Atg7, and Atg12 in membrane fractions from the brains of control, AD and DLB patients. Levels of Atg7 were significantly reduced in the brains of DLB patients. All semi-quantitative measurements were normalized to actin levels as a loading control. *p<0.05 compared to non-demented controls by one-way ANOVA with post-hoc Dunnett's test.

Immunohistochemical analysis showed moderate levels of mTor and Atg7 immunostaining in pyramidal neurons in control and AD cases (Figure 2A, B, D, E). In contrast, in DLB cases levels of neuronal mTor immunoreactivity were increased (Figure 2C, G), while the levels of neuronal Atg7 immunolabeling were reduced (Figure 2F, G). The increased levels of mTor and reduced Atg7 levels suggest there may be altered activation of the autophagy pathway in the brains of DLB patients. Consistent with this possibility, in DLB cases Cathepsin D-immunoreactive lysosomes of normal size were scant, and pyramidal cells contained enlarged lysosomes (Figure 2H–J, N) and increased levels of LC3 immunoreactivity (Figure 2K–M, O) compared to control cases.

**Figure 2:** Immunohistochemical analysis of the autophagy pathway in the brains of AD and DLB patients. Vibratome sections from the temporal cortex of non-demented controls, AD, and DLB patients were immunolabeled with antibodies against mTor, Atg7, Cathepsin D, and LC3, and imaged with a digital microscope. (A–C) Representative sections from control, AD and DLB brains immunolabeled with an antibody against mTor. (D–F) Representative sections from control, AD and DLB brains immunolabeled with an antibody against Atg7. (G) Semi-quantitative image analysis reveals a significant increase in mTor levels and a reduction in Atg7 levels in DLB patients compared to controls. (H–J) Representative sections from control, AD and DLB brains immunolabeled with an antibody against Cathepsin D. Pyramidal neurons in AD and DLB cases show enlarged Cathepsin D-immunoreactive lysosomes (arrows). (K–M) Representative sections from control, AD and DLB brains immunolabeled with an antibody against LC3. (N) Increased numbers of enlarged lysosomes (>1µm) in AD and DLB brains. (O) Semi-quantitative image analysis of LC3 immunoreactivity reveals increased LC3 levels in AD and DLB brains. Scale bar in panel (C) represents 20µm in all microscopy images. *p<0.05 compared to non-demented controls by one-way ANOVA with post-hoc Dunnett's test.

By immunoblot analysis, in the DLB cases there was an increase in immunoreactive bands representing monomeric and aggregated α-syn both in the cytosolic and membrane fractions (Figure S1A, B). In the AD, the levels of α-syn were slightly elevated compared to controls (Figure S1C). Consistent with the immunohistochemical analysis (Figure 2), by immunoblot, levels of LC3 and Cathepsin D in the membrane fractions were reduced in the DLB cases compared to non-demented controls (Figure S1A, C). In contrast, in the AD cases levels of Cathepsin D were elevated compared to non-demented controls (Figure S1A, C).

Compared to the unimpaired neurons in the control cases, in DLB brains, mTor and LC3 immunoreactivity were more abundant in neurons displaying α-syn accumulation (Figure 3A–L). In addition, in the DLB cases, LC3 immunoreactivity was occasionally associated with LBs (Figure 3J–L). Compared to control cases, these neurons also showed enlarged Cathepsin D-positive lysosomes (Figure 3M–R). Consistent with these observations, electron microscopy analysis revealed the presence of abundant and abnormal autophagosomes in these α-syn-positive neurons that were not detected in control cases (Figure 4A–D).

**Figure 3:** Double-immunolabeling analysis of autophagy markers and α-syn in the brains of patients with DLB. Vibratome sections from the temporal cortex of non-demented controls and DLB patients were immunolabeled with antibodies against α-syn, and co-labeled with antibodies against mTor, LC3 or Cathepsin D, and imaged with a laser scanning confocal microscope. (A–D) Double-immunolabeling analysis showing increased mTor immunoreactivity in neurons of DLB patients showing α-syn accumulation. (G–L) Double-immunolabeling analysis showing increased LC3 immunoreactivity in neurons of DLB patients showing α-syn accumulation. LC3 immunoreactivity was occasionally associated with LBs (arrows). (M–R) Double-immunolabeling analysis showing enlarged Cathepsin D-immunoreactive lysosomes (arrows) in neurons of DLB patients showing α-syn accumulation. Scale bar in panel (C) represents 15µm in panels A–L and 8µm in panels M–R.

**Figure 4:** Electron microscopic analysis of abnormal autophagosomes in patients with DLB and in α-syn tg mice. (A) Representative image from a non-demented control case showing normal neuronal lysosomes (arrow). (B–D) Abnormal autophagosomes and accumulation of electrodense deposits (arrows) in intraneuronal membrane-bound structures in the brains of patients with DLB. (E) Representative image from a non tg mouse brain showing normal neuronal lysosomes (arrow). (F–H) Abnormal autophagosome morphology and accumulation of electrodense deposits (arrows) in intraneuronal membrane-bound structures in the brains of α-syn tg mice. Scale bar in panel (C) represents 0.5µm in all panels.

### Alterations in Molecular Components of the Autophagy Pathway in A-Synuclein Transgenic Mice

Consistent with the studies in human brains, levels of mTor and p-mTor were increased in the mebrane fractions from brains of α-syn tg mice compared to non tg controls (Figure 5A–C). Moreover, levels of a molecular initiator of autophagy, Atg7, were reduced in α-syn tg brains compared to APP tg mice and non tg controls (Figure 5A, D). In contrast, other components of the autophagy pathway such as Atg5, Atg12 and Beclin-1 were not different among the non tg and tg mouse groups (Figure 5A, C, D).

**Figure 5:** Immunoblot analysis of the autophagy pathway in the brains of APP and α-syn tg mice. Brain homogenates from non tg, APP tg, and α-syn tg mice were separated into membrane and cytosolic fractions, and 20 µg of each sample was subjected to gel electrophoresis. Immunoblots were probed with antibodies against mTor, phosphorylated (p) mTor, Beclin-1, Atg5, Atg7, Atg12 and Actin. (A) Representative immunoblots of membrane fractions. (B) Representative immunoblots of cytosolic fractions. (C) Semi-quantitative analysis of levels of mTor, p-mTor, and Beclin-1 in membrane fractions from the brains of non tg, APP tg and α-syn tg mice. Levels of mTor were significantly increased in APP tg and α-syn tg brains. (D) Semi-quantitative analysis of levels of Atg5, Atg7, and Atg12 in membrane fractions from the brains of non tg, APP tg and α-syn tg mice. Levels of Atg7 were significantly reduced in the brains of α-syn tg mice. All semi-quantitative measurements were normalized to actin levels as a loading control. *p<0.05 compared to non tg controls by one-way ANOVA with post-hoc Dunnett's test.

In the non tg and APP tg mice, immunohistochemical analysis showed moderate levels of mTor and Atg7 immunostaining in pyramidal neurons in the neocortex (Figure 6A, B, D, E, G) and hippocampus (not shown). In contrast, in the α-syn tg mice levels of neuronal mTor immunoreactivity were increased, while the levels of neuronal Atg7 immunolabeling were reduced (Figure 6C, F, G). Compared to non tg control mice, in APP and α-syn tg mice pyramidal cells contained enlarged lysosomes (Figure 6H–J, N) and abnormal levels of LC3 immunoreactivity (Figure 6K–M, O). Abundant α-syn monomer and oligomers were detected in the membrane and cytosolic fractions of α-syn tg mice (Figure S2A, B). By immunoblot analysis, levels of LC3 in the membrane fraction were increased and Cathepsin D was reduced in the α-syn tg mice compared to non tg controls (Figure S2A, C). Compared to control mice, in the APP tg mice, levels of LC3 were elevated while levels of Cathepsin D were unchanged in the membrane fraction (Figure S2A, C). Double-labeling studies showed that mTor and LC3 were abundant in neurons displaying α-syn accumulation (Figure 7A–L). These neurons also showed the presence of enlarged Cathepsin D-positive lysosomes compared to non tg controls (Figure 7M–R). Electron microcopy analysis confirmed the presence of abundant and abnormal autophagosomes in these neurons (Figure 4E–H).

**Figure 6:** Immunohistochemical analysis of the autophagy pathway in the brains of APP and α-syn tg mice. Vibratome sections from the hippocampus of non tg, APP tg and α-syn tg mice were immunolabeled with antibodies against mTor, Atg7, Cathepsin D, or LC3, and imaged with a digital microscope. All images are from the temporal cortex. (A–C) Representative sections from non tg, APP tg and α-syn tg brains immunolabeled with an antibody against mTor. (D–F) Representative sections from non tg, APP tg and α-syn tg brains immunolabeled with an antibody against Atg7. (G) Semi-quantitative image analysis reveals a significant increase in mTor levels and a reduction in Atg7 levels in α-syn tg mice compared to non tg controls. (H–J) Representative sections from non tg, APP tg and α-syn tg brains immunolabeled with an antibody against Cathepsin D. Enlarged Cathepsin D-immunoreactive lysosomes (arrows) were detected in APP tg and α-syn tg mice. (K–M) Representative sections from non tg, APP tg and α-syn tg brains immunolabeled with an antibody against LC3. (N) Increased numbers of enlarged lysosomes (>1µm) in APP tg and α-syn tg mouse brains. (O) Semi-quantitative image analysis of LC3 immunoreactivity reveals increased LC3 levels in APP tg and α-syn tg brains. Scale bar in panel (C) represents 10µm in all microscopy images. *p<0.05 compared to non tg controls by one-way ANOVA with post-hoc Dunnett's test.

**Figure 7:** Double-immunolabeling analysis of autophagy and α-syn in the brains of α-syn tg mice. Vibratome sections from the brains of non tg and α-syn tg mice were immunolabeled with antibodies against α-syn, and co-labeled with antibodies against mTor, LC3 or Cathepsin D, and imaged with a laser scanning confocal microscope. All images are from the temporal cortex. (A–D) Double-immunolabeling analysis showing increased mTor immunoreactivity in α-syn-positive neurons in α-syn tg mice. (G–L) Double-immunolabeling analysis showing increased LC3 immunoreactivity in neurons of α-syn tg mice showing α-syn accumulation. (M–R) Double-immunolabeling analysis showing enlarged Cathepsin D-immunoreactive lysosomes (arrows) in neurons of α-syn tg mice showing α-syn accumulation. Scale bar in panel (C) represents 20µm in panels A–L and 10µm in panels M–R.

### Effects of Intra-Cerebral Infusion of mTor Inhibitor in A-Synuclein Transgenic Mice

Since alterations in the autophagy pathway in DLB and in α-syn tg mice might be in part related to increased levels of mTor, we investigated whether blocking mTor with rapamycin might promote α-syn clearance and be neuroprotective. Compared to vehicle-infused mice, in α-syn tg mice that received rapamycin treatment, α-syn accumulation in neuronal cell bodies and synapses was reduced and redistributed to the axons (Figure 8A–C, G). Moreover, compared to vehicle-treated α-syn tg mice, rapamycin treatment resulted in increased levels of LC3 (Figure 8D–G) and Cathepsin D (Figure 8H–J, N) immunoreactivity. Furthermore, this treatment ameliorated the dendritic pathology in the neocortex as reflected by image analysis of MAP2 immunolabeling of the neuropil (Figure 8K–N). By immunoblot analysis, compared to tg mice infused with vehicle alone, α-syn tg mice that received intra-cerebral infusions with rapamycin displayed reduced levels of α-syn in the membrane fraction with a concomitant increase in the lysosomal fraction (Figure 8O, P). In addition, rapamycin increased the levels of LC3 and Cathepsin D immunoreactivity (Figure 8O, P).

**Figure 8:** Immunohistochemical and immunoblot analysis of the effects of rapamycin treatment in α-syn tg mice. For panels A–M, vibratome sections from the hippocampus of non tg and α-syn tg mice were immunolabeled with antibodies against α-syn, LC3, Cathepsin D or MAP2 and imaged with a digital microscope. All images are from the temporal cortex. For panel O, brain homogenates from non tg and α-syn tg mice were separated into membrane and lysosomal fractions, and 20 µg of each sample was subjected to gel electrophoresis. (A–C) Representative sections from the brains of vehicle-treated non tg mice and vehicle- and Rapamycin-treated α-syn tg mice immunolabeled with an antibody against α-syn. (D–F) Representative sections from the brains of vehicle-treated non tg mice and vehicle- and Rapamycin-treated α-syn tg mice immunolabeled with an antibody against LC3. (G) Semi-quantitative image analysis showing reduced α-syn immunoreactivity and increased LC3 immunoreactivity in the hippocampus of α-syn tg mice treated with Rapamycin. (H–J) Representative sections from the brains of vehicle-treated non tg mice and vehicle- and Rapamycin-treated α-syn tg mice immunolabeled with an antibody against Cathepsin D. (K–M) Representative sections from the brains of vehicle-treated non tg mice and vehicle- and Rapamycin-treated α-syn tg mice immunolabeled with an antibody against MAP2. (N) Semi-quantitative image analysis showing increased Cathepsin D immunoreactivity in the hippocampus of α-syn tg mice treated with Rapamycin. Reduced levels of MAP2 in the hippocampus of vehicle-treated α-syn tg mice is rescued by Rapamycin treatment. (O) Representative immunoblot analysis of membrane and lysosomal fractions probed with antibodies against α-syn, LC3, and Cathepsin D. (P) Semi-quantitative image analysis of immunoblots showing redistribution of α-syn from membrane to lysosomal fractions and an associated increase in LC3 and Cathepsin D levels. All semi-quantitative measurements were normalized to actin levels as a loading control. Scale bar in panel (C) represents 40µm in panels A–C, 20µm in panels D–E and H–J, and 10µm in panels K–M. *p<0.05 compared to vehicle-treated non tg controls by one-way ANOVA with post-hoc Dunnett's test. #p<0.05 compared to vehicle-treated α-syn tg mice by one-way ANOVA with post-hoc Tukey-Kramer test.

Taken together, these results support the possibility that alterations in the autophagy pathway and more specifically in mTor and Atg7 are associated with accumulation of α-syn and neurodegeneration in DLB cases and α-syn tg models, and activation of autophagy with rapamycin can revert this effect.

### Lentivirus Delivery of Atg7 Rescues α-Synuclein Accumulation and Neuronal Deficits in Transgenic Mice

Since in addition to the increase in mTor, we also observed a reduction in Atg7 levels in DLB and α-syn tg mice, we sought to determine whether viral-mediated delivery of Atg7 might also promote α-syn clearance and rescue neurodegenerative deficits in α-syn tg mice. For this purpose, we delivered the Atg7 lentivirus via stereotaxic injection to the temporal cortex and hippocampus of non tg and α-syn tg mice [55].

Compared to non tg and α-syn tg mice treated with the LV-control (Figure 9A–D, G) delivery of LV-Atg7 resulted in increased expression in Atg7 in pyramidal neurons in the hippocampus and in areas adjacent to the injection track in the neocortex (Figure 9E–G). Atg7 immunostaining was localized primarily to the neuronal perykaria surrounding the injection track with some extension to the apical dendrites (Figure 9E). Compared to non tg mice (Figure 9H, I), α-syn tg mice injected with the LV-control contained abundant intracellular aggregates of α-syn (Figure 9J, K); in contrast, following LV-Atg7 injection, there was a considerable reduction in the intra-neuronal α-syn accumulation in the areas adjacent to the injection track (Figure 9L–N).

**Figure 9:** Immunohistochemical analysis of the effects of LV-Atg7 treatment in α-syn tg mice. For panels A–M, vibratome sections from non tg and α-syn tg mice that received LV injections into the cortex and hippocampus were immunolabeled with antibodies against Atg7 or α-syn and imaged with a digital microscope. Panels A′–M′ represent higher-power images from the hippocampus of the corresponding low-power panels in panels A–M. For panels O–T, effects of rapamycin treatment on α-syn accumulation, autophagy and neuronal integrity in the brains of α-syn tg mice. For panels A–M, vibratome sections from the hippocampus of non tg and α-syn tg mice were immunolabeled with an antibody against MAP2 and imaged with a laser scanning confocal microscope, and images were obtained from the temporal cortex. (A–F) Representative sections from the brains of non tg (A, B) and α-syn tg mice (C–F) that received injections with LV-control (A–D) or LV-Atg7 (E, F) and were immunolabeled with an antibody against Atg7. Images show sections from the hemisphere ipsilateral (ipsi) or contralateral (contra) to the sites of injection. (G) Semi-quantitative image analysis of Atg7 immunoreactivity in non tg and α-syn tg mice show increased Atg7 levels ipsilateral to the injection sites in the brains of animals that received LV-Atg7. (H–M) Representative sections from the brains of non tg (H, I) and α-syn tg mice (J–M) that received injections with LV-control (H–K) or LV-Atg7 (L, M) and were immunolabeled with an antibody against α-syn. Images show sections from the hemisphere ipsilateral (ipsi) or contralateral (contra) to the sites of injection. (N) Semi-quantitative image analysis of α-syn immunoreactivity in non tg and α-syn tg mice show reduced α-syn levels ipsilateral to the injection sites in the brains of α-syn tg mice that received LV-Atg7 injections. (O–T) Representative sections from the brains of non tg (O, P) and α-syn tg mice (Q–T) that received injections with LV-control (O–R) or LV-Atg7 (S, T) and were immunolabeled with an antibody against MAP2. Images show sections from the hemisphere ipsilateral (ipsi) or contralateral (contra) to the sites of injection. (U) Semi-quantitative image analysis of MAP2 immunoreactivity in non tg and α-syn tg mice shows a recovery of MAP2 levels ipsilateral to the injection sites in the brains of α-syn tg mice that received LV-Atg7 injections. Scale bar in panel (F) represents 0.1mm in panels A–F and H–M, 20µm in panels A′–F′ and H′–M′, and 10µm in panels O–T. *p<0.05 compared to LV-control-treated non tg controls by one-way ANOVA with post-hoc Dunnett's test. #p<0.05 compared to LV-control-treated α-syn tg mice by one-way ANOVA with post-hoc Tukey-Kramer test.

Concomitant with the reduction in α-syn accumulation, analysis of the dendritic marker MAP2 showed an increase in the percent area of the neuropil covered by dendrites in α-syn tg mice that received the LV-Atg7 (Figure 9O–U), supporting the possibility that the reduction of α-syn accumulation in the LV-Atg7-treated animals ameliorated the structural damage to neurons of α-syn tg mice. Importantly, no significant deleterious effects on neuronal or synapto-dendritic content were observed in non tg mice that received injections with LV-Atg7 (not shown). Together, these data suggest that delivery of LV-Atg7 to the α-syn tg mice reduced the accumulation of α-syn and related neuronal pathology by inducing a physiological autophagic response.

### Overexpression of Atg7 in an *In Vitro* Model Reduces α-Synuclein Accumulation, while Atg7 Knockdown Exacerbates Autophagic Deficits and α-Synuclein Accumulation

To further confirm the effects of LV-Atg7 in activating autophagy and promoting α-syn clearance, we utilized a neuronal cell model to study autophagy in the presence of α-syn accumulation [42]. For this purpose, B103 neuronal cells were infected with lentivirus expressing an LC3-GFP fusion protein and co-infected with LV-control or LV-αsyn. The LC3-GFP is a marker for autophagy activation, and increased LC3-GFP fluorescence indicates increased autophagic activity. These cells were then infected with either LV-Atg7 or a virus encoding an shRNA against Atg7 or a control shRNA against luciferase. Immunocytochemical analysis demonstrated that compared to controls (Figure S3A) levels of Atg7 were higher in LV-Atg7-infected cells (Figure S3B), while baseline levels of Atg7 were reduced by the LV-shAtg7 (Figure S3C). Consistent with the immunocytochemical analysis, western blot confirmed the expression and knockdown of Atg7 in the LV infected neuronal cell line (Figure S3D).

Immunolabeling studies with an antibody against α-syn demonstrated that compared to controls (Figure 10A, F) and LV-Atg7 infected cells (Figure 10B, F), there was an increase in expression of α-syn in LV-αsyn infected cells (Figure 10C, F). Infection with LV-Atg7 resulted in increased numbers of LC3-GFP grains per cell, consistent with an activation of autophagy (Figure 10B, E). In cells co-infected with LV-αsyn, co-expression of Atg7 also resulted in significant activation of autophagy (Figure 10D, E) and a reduction in α-syn accumulation (Figure 10D, F). Similar experiments with LV-βsyn and LV-Atg7 showed no reduction in levels of β-syn, indicating that Atg7 expression specifically reduced the accumulated levels of α-syn (data not shown).

**Figure 10:** Immunocytochemical analysis of the effects of Atg7 over-expression or knockdown in a neuronal cell model. For Atg7 overexpression, B103 neuronal cells on coverslips and infected with a lentivirus expressing LC3-GFP in combination with empty LV-control, LV-Atg7, or LV-α-syn. For Atg7 knockdown, B103 neuronal cells on coverslips were infected with a lentivirus expressing LC3-GFP in combination with empty LV-shControl, LV-shAtg, or LV-αsyn. Cells were fixed and immunolabled with an antibody against α-syn and imaged with a laser scanning confocal microscope. In each set of 3 panels, the upper left panel depicts GFP fluorescence, the upper right panel depicts α-syn immunolabeling, and the lower panel depicts the merged image. (A–D) Representative images showing GFP fluorescence (marker of LC3 localization) and α-syn immunoreactivity in B103 cells infected with LV-control (A), LV-Atg7 (B), LV-αsyn (C) or LV-Atg7+LV-αsyn (D). (E) Semi-quantitative analysis of LC3-GFP positive punctae shows an increase in LC3 in cultures infected with LV-Atg7 or LV-α-syn alone or in combination. (F) Semi-quantitative analysis of α-syn immunoreactivity reveals a reduction in α-syn levels in cultures co-infected with LV-Atg7 and LV-αsyn. (G–J) Representative images showing GFP fluorescence (marker of LC3 localization) and α-syn immunoreactivity in B103 cells infected with LV-shControl (G), LV-shAtg7 (H), LV-αsyn (I) or LV-shAtg7+LV-αsyn (J). (K) Semi-quantitative analysis of LC3-GFP positive punctae shows a reduction in LC3 in cultures infected with LV-shAtg7 alone or in combination with LV-αsyn. (L) Semi-quantitative analysis of α-syn immunoreactivity reveals an increase in α-syn levels in cultures co-infected with LV-shAtg7 and LV-αsyn. Scale bar in large panel in (D) represents 15µm in all small panels and 10µm in all large panels. *p<0.05 compared to LV-control-treated cultures by one-way ANOVA with post-hoc Dunnett's test. #p<0.05 compared to LV-αsyn-treated cultures by one-way ANOVA with post-hoc Tukey-Kramer test.

In contrast, compared to LV-shControl (Figure 10G, K), when neuronal cells were infected with the LV-shAtg7, levels of LC3-GFP were reduced (Figure 10H, K). Similar effects were observed in neuronal cells co-infected with LV-shAtg7 and LV-αsyn (Figure 10I–K). Moreover, compared LV-shControl (Figure 10G, I, L), in cells infected with LV-shAtg7, the levels of α-syn accumulation were increased (Figure 10J, L). Taken together, these results support the possibility that activating the autophagy pathway with rapamycin or with viral delivery of Atg7 might reduce the accumulation of α-syn and rescue the associated neurodegenerative alterations.

## Discussion

Recent evidence in cell-based models of PD-like pathology indicate that alterations in lysosomal functioning and autophagy might participate in the mechanisms of α-syn-mediated neurodegeneration [23], [29], [35], [36], [37], [38], [39]. However it was unclear which molecular components of the autophagy pathway might be dysregulated in the brains of patients with DLB/PD and in α-syn tg models. For the present study we chose investigate potential alterations in components of autophagy in DLB cases (rather than pure PD) because after AD, these cases represent the most common form of dementia and movement disorders in the aging population and display widespread cortical and subcortical pathology.

Remarkably, we found that in DLB cases and in α-syn tg mice levels of mTor were elevated and Atg7 expression was reduced. mTor and LC3 was co-localized with neurons displaying α-syn accumulation and neurodegenerative changes. This is of interest because it provides a potential alternative explanation for the molecular alterations in autophagy in sporadic forms of LBD. mTor and Atg7 are early initiators of the macroautophagy pathway. Inhibition of mTor by nutrient reduction or by activation of PI3K results in activation of the Atg kinase 1 that in turn phosphorylates Atgs that participate in the AV formation [71], [72], [73].

The mechanisms through which increased mTor and reduced Atg7 might participate in the neuropathology of DLB are not completely clear. However, such alterations are predicted to result in deficient initiation of the autophagy process. This in turn might result in progressive accumulation of α-syn aggregates that further interfere with the fusion of lysosomes and formation of autophagosomes, as has been suggested by other studies [23], [40], [41]. This may then lead to the formation of enlarged and atypical AV-like structures [42]. Supporting this possibility, the present study also showed that the cortical neurons in DLB cases and in α-syn tg mice contained enlarged lysosomes and autophagosomes similar to those described in AD [33]. The formation of such abnormal AV-like structures in DLB and α-syn tg mice is consistent with recent reports in neuronal cells lines overexpressing α-syn [42]. These cells show the presence of granular α-syn aggregates that co-localize with abnormally enlarged LC3-positive structures [42]. The accumulation of α-syn and the neurodegenerative phenotype in neuronal cells was reverted by activation of the autophagy pathway with a gene therapy approach delivering Beclin-1 with a lentivirus [42] or with rapamycin [42], [74], [75]. In agreement with these findings, the present study showed *in vivo* that infusion of rapamycin or injection of LV-Atg7 into the brains of tg mice reduced the accumulation of α-syn and was neuroprotective. This is consistent with previous *in vivo* studies showing that rapamycin is neuroprotective in models of neurodegeneration [76], [77], AD [78] and Huntington's Disease [79], [80]. Moreover, a recent study showed that blocking mTor by overexpression of the translation inhibitor Thor (4E-BP) can reduce the pathologic features in PD models, including degeneration of dopaminergic neurons in Drosophila [81]. Moreover, rapamycin activates *in vivo* 4E-BP and rapamycin is also capable of ameliorating the pathology associated with mutations in other PD associated genes such as Pink1 and parkin [81].

In familial types of parkinsonism, mutant forms of α-syn [23] have been shown to disrupt lysosomal clearance by blocking CMA. Further supporting a role for lysosomal dysfunction in DLB and PD, recent studies have shown that in lysosomal storage disorders such as Gaucher disease [43], [44] and Niemann-Pick disease [45], there is increased predisposition to develop parkinsonism and α-syn accumulation. Other animal studies in models of PD, such as in animals exposed to the neurotoxin 1-methyl-4-phenyl-1,2,3,6-tetrahydro-pyridine (MPTP), have also revealed autophagic dysfunction associated with alterations in signal transduction pathways [82]. In addition, increased susceptibility to develop PD appears to be associated with polymorphisms in lysosomal genes such as those associated with Gaucher disease and Niemann-Pick disease. Moreover, recent studies have shown that reduced Cathepsin D expression results in α-syn accumulation and degeneration of the dopaminergic system in experimental models and in patients with PD [83]. Cathepsin D is now considered one of the main lysosomal enzymes involved in α-syn degradation [84] and overexpression of Cathepsin D reduces the pathology associated with α-syn accumulation [85].

Selective alterations in molecular components of the autophagy pathway might result in degeneration of specific neuronal populations in neurological disorders. For example, previous studies have shown that in sporadic AD there is a profound reduction in the levels of Beclin-1 [34], while the neurodegenerative process in familial forms of fronto-temporal dementia and ALS has been linked to mutations in charged multivesicular body protein-2B (CHMP2B) [86], [87], [88], and in Huntington's Disease polyglutamate aggregates trap mTor and disrupt autophagy [80].

The mechanisms through which levels of mTor might be upregulated and Atg7 downregulated in DLB and α-syn tg mice are not completely clear. However, targeted reduction of autophagy genes including Atg7 results in behavioral defects, including abnormal limb-clasping reflexes and a reduction in coordinated movement, and died within 28 weeks of birth. Furthermore, Atg7 deficiency results in neurodegeneration of the cerebral and cerebellar cortices [89].

In conclusion, this study supports the notion that selective molecular alterations in the autophagy pathway and more specifically in mTor and Atg7 are associated with DLB and α-syn tg models and supports the possibility that modulators of the autophagy pathway might have potential therapeutic effects.

## Supporting Information

Figure S1 Immunoblot analysis of α-syn levels and lysosomal markers in the brains of AD and DLB patients. Brain homogenates from the temporal cortex of non-demented controls, AD, and DLB patients were separated into membrane and cytosolic fractions, and 20 µg of each sample was subjected to gel electrophoresis. Immunoblots were probed with antibodies against α-syn, Cathepsin D, LC3 and Actin. (A) Representative immunoblots of membrane fractions. (B) Representative immunoblots of cytosolic fractions. (C) Semi-quantitative analysis of levels of α-syn, Cathepsin D and LC3 in membrane fractions from the brains of control, AD and DLB patients. Levels of Cathepsin D were increased in the brains of AD patients but reduced in the brains of DLB patients, while levels of LC3 were increased in the brains of both AD and DLB patients. All semi-quantitative measurements were normalized to actin levels as a loading control. *p<0.05 compared to non-demented controls by one-way ANOVA with post-hoc Dunnett's test.
(0.41 MB TIF)

Figure S2 Immunoblot analysis of α-syn levels and lysosomal markers in the brains of APP tg and α-syn tg mice. Brain homogenates from non tg, APP tg, and α-syn tg mice were separated into membrane and cytosolic fractions, and 20 µg of each sample was subjected to gel electrophoresis. Immunoblots were probed with antibodies against α-syn, Cathepsin D, LC3 and Actin. (A) Representative immunoblots of membrane fractions. (B) Representative immunoblots of cytosolic fractions. (C) Semi-quantitative analysis of levels of α-syn, Cathepsin D and LC3 in membrane fractions from the brains of non tg, APP tg and α-syn tg mice. Levels of Cathepsin D were significantly reduced in α-syn tg brains, while levels of LC3 were increased in the brains of APP tg and α-syn tg mice. All semi-quantitative measurements were normalized to actin levels as a loading control. *p<0.05 compared to non tg controls by one-way ANOVA with post-hoc Dunnett's test.
(0.33 MB TIF)

Figure S3 Immunocytochemical and immunoblot characterization of lentivirus-mediated Atg7 over-expression and knockdown in a neuronal cell line. B103 neuronal cells on coverslips were infected with LV-Atg7 or LV-shAtg7, followed by fixation and immunolabeling with an antibody against Atg7, or lysis and immunoblot analysis with antibodies against Atg7 or Actin. (A) Representative image of endogenous Atg7 immunoreactivity in cells infected with empty LV-control. (B) Representative image showing increased Atg7 immunoreactivity in cells infected with LV-Atg7. (C) Representative image showing reduced Atg7 immunoreactivity in cells infected with LV-shAtg7. (D) Representative immunoblot showing Atg7 levels in cells infected with LV-Atg7 or LV-shAtg7. Scale bar in panel (C) represents 40µm in all microscopy images.
(0.80 MB TIF)
